# Ulinastatin as an Adjuvant Therapy to Restricting Volumes of Resuscitation Fluid Strategy for Patients with Septic Shock after Initial Management

**DOI:** 10.1155/2021/4231454

**Published:** 2021-06-16

**Authors:** Rensong Dong, Xi Zhang, Zhi Zhao

**Affiliations:** ^1^Department of Pharmacy, The Second Hospital of Hebei Medical University, Shijiazhuang, China; ^2^Department of Neurology, The Second Hospital of Hebei Medical University, Shijiazhuang, China

## Abstract

Septic shock is the most serious complication of sepsis, leading to unacceptably high morbidity and mortality worldwide. Fluid resuscitation using crystalloids has become the mainstay of early and aggressive treatment of severe sepsis and septic shock, while increased daily fluid balances from day 2 until day 7 have been related with increased mortality. Recently, pharmacological management has been recommended to combine with appropriate fluid resuscitation for the treatment of septic shock. In this study, we compared the clinical efficacy of restricting volumes of resuscitation fluid strategy with or without intravenous infusion of ulinastatin (UTI) in treating patients with septic shock and additionally examined the patient's changes of the extravascular lung water index (EVLWI), pulmonary vascular permeability index (PVPI), systemic vascular resistance index (SVRI), cardiac function, lactic acid (LA) level, coagulation function, and renal function. The study included 182 patients with septic shock, among which 89 patients had undergone restricting volumes of resuscitation fluid strategy with intravenous infusion of UTI and 93 patients had undergone restricting volumes of resuscitation fluid strategy alone. It was found that patients with septic shock after restricting volumes of resuscitation fluid strategy with intravenous infusion of UTI showed an increased SVRI concomitant with declined PVPI and EVLWI, increased mean artery pressure (MAP), cardiac output (CO), left ventricular ejection fraction (LVEF), stroke volume (SV), and heart rate (HR), declined levels of cardiac troponin I (cTnI), N-terminal pro-B-type natriuretic peptide (NT-proBNP), and C-reactive protein (CRP), reduced LA level along with shortened prothrombin time (PT) and partially activated thrombin time (PATT), and decreased levels of blood urea nitrogen (BUN), creatinine (Cr), and uric acid (UA) when comparable to those after restricting volumes of resuscitation fluid strategy alone (*P* < 0.05). We also observed fewer scores of the Acute Physiology and Chronic Health Evaluation (APACHE II) and the sequential organ failure assessment (SOFA) in patients undergoing restricting volumes of resuscitation fluid strategy with intravenous infusion of UTI than those undergoing restricting volumes of resuscitation fluid strategy alone (*P* < 0.05). According to the above data, it is concluded that UTI as an adjuvant therapy for restricting volumes of resuscitation fluid strategy in treating septic shock may decrease the LA level, attenuate the inflammatory response, reduce vascular permeability, prevent pulmonary edema, and restore cardiac and renal functions.

## 1. Introduction

Sepsis is considered as a process of infection in systemic inflammatory response syndrome. Nowadays, sepsis has been redefined as life-threatening organ dysfunction induced by a prolonged imbalance of innate immune response to infection [1]. Septic shock is the severest condition following sepsis and exhibits a poor prognostic outcome with a mortality rate of up to 50%, which is a leading reason for admission into the intensive care unit (ICU) [2]. Sepsis is mainly caused by pulmonary infection and abdominal infection [3]. The incidence of sepsis is higher in males than in females [4], which may relate to the protective effect of estrogen on immune function and cardiovascular function, since there is a negative correlation between cell-mediated immune response and androgen [5]. Despite its mortality has been decreased over the years due to the improvements of ICU and therapeutic strategies, sepsis shock is still one of the major medical problems in the world, especially in developed countries, resulting in a large consumption of medical resources [6–8].

The pathogenesis of sepsis is very complex and remains unclear, which leads to limited treatment [9]. Since sepsis and septic shock are related to immunosuppression, the supplement of immunological factors might be an effective therapy, but the guidelines (Surviving Sepsis Campaign Guidelines for Management of Sepsis and Septic Shock) still do not recommend intravenous immunoglobulin (IG) in septic patients [10]. The administration of appropriate intravenous antibiotics probably is made rapidly within the first hour after sepsis or septic shock is diagnosed; each hour delay is associated with increased mortality [11, 12]. In addition to antibiotics, the intravenous fluid resuscitation is the most common intervention in sepsis therapy, especially for patients in the ICU [13], and the preferred resuscitation fluid is crystalloid [14, 15]. The organ edema and organ dysfunction caused by excessive fluid infusion were reported in some clinical data [16–18]. Ulinastatin (UTI) is a protease inhibitor with more extensive inhibitory activity compared with the others, which can inhibit trypsin and polymorphonuclear leukocyte elastase which is considered to be one of the most destructive enzymes in sepsis [19]. Early intravenous UTI was related to the reduced mortality of patients with severe sepsis through improving organ dysfunction, which is reported in a randomized controlled trial [20]. In this study, we compared the clinical efficacy of restricting volumes of resuscitation fluid strategy with or without intravenous infusion of UTI in treating patients with septic shock and additionally examined the patient's changes of the extravascular lung water index (EVLWI), pulmonary vascular permeability index (PVPI), systemic vascular resistance index (SVRI), cardiac function, coagulation function, and renal function.

## 2. Materials and Methods

### 2.1. Study Design and Population

This investigation is a retrospective cohort study of 182 patients with septic shock admitted to the ICU of our hospital from December 2018 to December 2020. All 182 patients fulfilled the International Guidelines for Management of Sepsis and Septic Shock (2016) [10] within the previous 24 h: evidence of infection symbols; presence of systemic inflammatory response; systolic pressure < 90 mmHg (1 mmHg = 0.133 kPa); poor tissue perfusion, such as oliguria (<30 mL/h) more than 1 h; or acute neurological disorders. Patients were excluded for the following reasons: (1) treatment with antibiotics, hormones, or gamma globulin in the past three months; (2) a history of congestive heart failure with an LVEF < 40%; (3) requirement for extracorporeal membrane oxygenation or the use of a ventricular assist device or developed septic shock at an outside hospital requiring vasopressor and fluid management prior to transfer; (4) complication with metabolic diseases or malignant tumors; (5) severe liver and kidney dysfunction; (6) hematological or immune system diseases; (7) cognitive impairment or mental disease; (8) poor compliance to the treatment protocol; (9) confirmed or suspected pregnancy and lactation; (10) allergic to UTI.

### 2.2. Fluid Resuscitation Protocols and Intravenous Infusion of UTI

All included patients were given conventional antishock and anti-infection treatments, and vital signs were monitored after admission. For anti-infection treatments, third-generation cephalosporin combined with vancomycin or carbapenem antibiotics was used for the treatment of septic shock with unknown reasons, and the antibiotics were changed according to the experimental results of the blood culture later. The vital signs of patients were monitored with supplemental oxygen to maintain SpO_2_   >  92%. Antishock treatments were performed using crystalloid or colloid solutions based on the ratio of 2 : 1. The patients were supplemented by initial resuscitation fluid with Ringer's solution at a total volume of 500–1000 ml within 1 h to maintain mean arterial pressure (MAP) between 50 and 60 mmHg and urine discharge 0.5–1.0 ml/kg/h. Continued fluid boluses (at a maintenance <3000 ml per day) via the infusion pump were given in case of severe hypoperfusion defined as either plasma concentration of lactate of at least 4 mmol/L or MAP below 50 mmHg in spite of the infusion of norepinephrine. UTI (200,000 IU/day, Techpool Bio-Pharma Co., Ltd, H19900134, Guangdong, China) was dissolved in normal saline and intravenously injected or pumped into the patients for consecutive 7 days.

### 2.3. Outcome Measures

Each patient was scored using the Acute Physiology and Chronic Health Evaluation (APACHE II) [21] and the sequential organ failure assessment (SOFA) [22]. SVRI, PVPI, and EVLWI were monitored by using the pulse indicator continuous cardiac output (PiCCO) instrument. In detail, a certain amount of cold saline was injected from the central vein to the receiving end of the PiCCO catheter through the superior vena cava, right atrium, right ventricle, pulmonary artery, extravascular lung water, pulmonary vein, left atrium, left ventricle, ascending aorta, abdominal aorta, and femoral artery. Cardiac functions were evaluated by analyzing mean artery pressure (MAP), heart rate (HR), cardiac output (CO), left ventricular ejection fraction (LVEF), stroke volume (SV), plasma levels of cardiac troponin I (cTnI), N-terminal pro-B-type natriuretic peptide (NT-proBNP), and C-reactive protein (CRP). Fasting venous blood was collected before treatment and at 7 days after treatment. The plasma concentration of cTnT was examined by immunoassay (Elecsys 1020, Boehringer Mannheim Diagnostics, Germany). The plasma NT-proBNP level was ascertained using a high-sensitivity immunoradiometric assay (Shionogi, Osaka, Japan). The plasma concentrations of CRP, blood urea nitrogen (BUN), creatinine (Cr), and uric acid (UA) were determined using BeckmannAssay360 (Beckman, Bera, CA, USA). The serum level of lactic acid (LA), prothrombin time (PT), and partially activated thrombin time (PATT) were determined. The mortality was recorded after 7 days of treatment.

### 2.4. Data Processing

SPSS 22.0 software was employed to perform data management and analysis. Continuous variables are displayed by mean ± standard deviation and analyzed by the *t*-test. Categorical variables are expressed as proportions and analyzed using the chi-square test. A possibility of significant difference is shown as *P* < 0.05.

## 3. Results

### 3.1. Baseline Variables of Study Participants

The study included 182 patients with septic shock, and they were split into the fluid restriction group (*n* = 89) and fluid restriction + UTI treatment group (*n* = 93) according to restricting volumes of resuscitation fluid strategy with or without intravenous infusion of UTI. As shown in Table 1, the fluid restriction group and fluid restriction + UTI treatment group were comparable since no significant difference was observed between the two groups with regard to sex, age, and source of sepsis (*P* > 0.05).

### 3.2. The Changes of SVRI, PVPI, and EVLWI in Patients with Septic Shock after Restricting Volumes of Resuscitation Fluid Strategy with or without Intravenous Infusion of UTI

Sepsis usually causes dysfunction of pulmonary microvascular endothelial cells, resulting in pulmonary edema. In this part, SVRI, PVPI, and EVLWI were examined in patients with septic shock after restricting volumes of resuscitation fluid strategy with or without intravenous infusion of UTI. There was a slight difference in SVRI, PVPI, and EVLWI between the fluid restriction group and fluid restriction + UTI treatment group at admission (*P* > 0.05). After treatment, patients with septic shock exhibited an increased SVRI concomitant with declined PVPI and EVLWI (*P* < 0.05). More importantly, patients with septic shock after restricting volumes of resuscitation fluid strategy with intravenous infusion of UTI showed an increased SVRI concomitant with declined PVPI and EVLWI when comparable to those after restricting volumes of resuscitation fluid strategy alone (*P* < 0.05, Table 2). It was revealed that adjuvant injection of UTI to restricting volumes of resuscitation fluid strategy may reduce vascular permeability and prevent patients with septic shock from subsequent pulmonary edema.

### 3.3. The Cardiac Function of Patients with Septic Shock after Restricting Volumes of Resuscitation Fluid Strategy with or without Intravenous Infusion of UTI

It is clear that cardiac dysfunction, as evidenced by biventricular dilatation and reduced LVEF, is present in most patients with severe sepsis and septic shock. To reflect the patient's cardiac function, MAP, CO, SV, LVEF, and HR were examined before and after restricting volumes of resuscitation fluid strategy with or without intravenous infusion of UTI. There was little difference with regard to CO, LVEF, and SV between the fluid restriction group and fluid restriction + UTI treatment group at admission (*P* > 0.05). After treatment, patients with septic shock displayed elevated MAP, CO, SV, LVEF, and HR (*P* < 0.05). It was found that patients with septic shock after restricting volumes of resuscitation fluid strategy with intravenous infusion of UTI showed increased MAP, CO, SV, LVEF, and HR when comparable to those after restricting volumes of resuscitation fluid strategy alone (*P* < 0.05, Table 3). Furthermore, the plasma levels of cTnI, NT-proBNP, and CRP were examined in patients with septic shock to reflect cardiac function before and after restricting volumes of resuscitation fluid strategy with or without intravenous infusion of UTI. No significant difference on the plasma levels of cTnI, NT-proBNP, and CRP was observed before treatment (*P* < 0.05). The patients in both fluid restriction group and fluid restriction + UTI treatment group had declined plasma levels of cTnI, NT-proBNP, and CRP after treatment (*P* < 0.05). Besides, the plasma levels of cTnI, NT-proBNP, and CRP were lower in patients after restricting volumes of resuscitation fluid strategy with intravenous infusion of UTI than in those after restricting volumes of resuscitation fluid strategy alone (*P* < 0.05, Figure 1). It was revealed that adjuvant injection of UTI to restricting volumes of resuscitation fluid strategy may restore cardiac function.

### 3.4. The LA and Coagulation Function of Patients with Septic Shock after Restricting Volumes of Resuscitation Fluid Strategy with or without Intravenous Infusion of UTI

No significant difference on the LA level, PT, and PATT was observed prior to treatment (*P* > 0.05). The patients in the fluid restriction group and fluid restriction + UTI treatment group showed a decreased LA level along with prolonged PT and PATT after treatment (*P* < 0.05). Besides, the LA level was lower, but PT and PATT were shorter in patients after restricting volumes of resuscitation fluid strategy with intravenous infusion of UTI than in those after restricting volumes of resuscitation fluid strategy alone (*P* < 0.05, Table 4), suggesting that adjuvant injection of UTI to restricting volumes of resuscitation fluid strategy could maintain coagulation function of patients with septic shock.

### 3.5. The Renal Function of Patients with Septic Shock after Restricting Volumes of Resuscitation Fluid Strategy with or without Intravenous Infusion of UTI

Acute renal failure commonly occurs with severe sepsis and is associated with high mortality. To evaluate the renal function, the volume of 24 h urine and the levels of BUN, Cr, and UA were examined in patients with septic shock before and after restricting volumes of resuscitation fluid strategy with or without intravenous infusion of UTI. There was no remarkable difference in terms of the volume of 24 h urine and the levels of BUN, Cr, and UA between the fluid restriction group and fluid restriction + UTI treatment group (*P* > 0.05). The patients in both fluid restriction group and fluid restriction + UTI treatment group had increased volume of 24 h urine and declined levels of BUN, Cr, and UA after treatment (*P* < 0.05). We also found that, except the volume of 24 h urine, reduced levels of BUN, Cr, and UA were determined in the fluid restriction + UTI treatment group compared with the fluid restriction group (*P* < 0.05, Figure 2).

### 3.6. Clinical Efficacy and Safety of Restricting Volumes of Resuscitation Fluid Strategy with or without Intravenous Infusion of UTI

At last, we compared the clinical efficacy and safety between restricting volumes of resuscitation fluid strategy with or without intravenous infusion of UTI. As shown in Table 5, there was a slight difference concerning APACHE II and SOFA scores between fluid restriction + UTI treatment and fluid restriction groups before treatment; the two groups had fewer APACHE II and SOFA scores after treatment (*P* < 0.05). We also observed fewer APACHE II and SOFA scores in the fluid restriction + UTI treatment group than the fluid restriction group. After treatment, the mortalities of the two groups did not differ (*P* > 0.05, Table 6).

## 4. Discussion

At the very beginning, the term sepsis was thought to be a process of flesh decay, which could be traced back to Hippocrates [23]. In 2016, the term sepsis was developed as organ dysfunction caused by host's maladjustment to infection, with high incidence and mortality, and septic shock was defined as a subtype of sepsis with severe circulatory, cellular, and metabolic abnormalities [6, 24]. Sepsis remains the main cause of morbidity and mortality all over the world, with significant regional differences, and it is more commonly seen in sub-Saharan, Oceania, South Asia, East Asia, and Southeast Asia, which might be related to lower medical conditions [8, 25].

The early fluid resuscitation is the essential treatment to patients with septic shock or increased blood LA level, and the initial fluid resuscitation should be done within 3 hours after the diagnosis of sepsis. At least 30 ml/kg of intravenous crystalloids is recommended initially [26]. However, few literature studies are available to support this proposal [27]. Some studies including experiment, observation, and randomized clinical trial showed that restricting volumes of resuscitation fluid strategy achieved much better outcomes [28–30]. The aim of this study is to investigate whether restricting volumes of resuscitation fluid strategy combined with UTI administration has a positive impact on cardiovascular function, coagulation index, and blood LA level. UTI is a serine protease inhibitor with anti-inflammatory effect [31], which was approved to reduce the mortality in the treatment of severe sepsis of randomized clinical trials [32], and also found a decrease of mortality in patients with severe sepsis treated with intravenous administration of UTI in combination with alpha thymosin [33–35]. Hemodynamic monitoring is very important for the diagnosis and treatment of critical patients. A research found that the decline of angiopoietin-2 (Ang-2) and EVLWI in sepsis patients was complicated by acute respiratory distress syndrome (ARDS), which was significantly related to the reduced death rate at 24 hours after admission [36]; this finding was similar with another study describing that, after 72 hours of treatment of high-volume hemofiltration (HVHF), the increase of EVLWI and PVPI was negatively correlated with the survival rate of patients with septic shock [37]. Vasoplegia is characterized by an abnormally low systemic vascular resistance index (SVRI), which was commonly seen in septic, neurogenic, and anaphylactic shock [38, 39]. A previous study showed that the SVRI was significantly reduced in the nonsurvivors than in the survivors in the septic shock after treatment for 24 hours, which suggested that the SVRI is associated with mortality [40]. This study found that, after 7 days of treatment, patients with septic shock after restricting volumes of resuscitation fluid strategy with intravenous infusion of UTI showed an increased SVRI concomitant with declined PVPI and EVLWI when comparable to those after restricting volumes of resuscitation fluid strategy alone.

MAP, CO, SV, LVEF, and HR are usually used to evaluate cardiac function, which were approved as close relevance with mortality in cardiogenic shock [41]. In this analysis, we found that patients with septic shock after restricting volumes of resuscitation fluid strategy with intravenous infusion of UTI showed increased MAP, CO, SV, LVEF, and HR when comparable to those after restricting volumes of resuscitation fluid strategy alone. cTnI, a marker of subclinical myocardial damage, has been reported as a predictor of thromboembolic events in patients with atrial fibrillation [42]. NT-proBNP is a new biomarker of cardiac function and heart failure and has become available as a clinical laboratory test in clinics [43]. Peak CRP is an independent predictor of left ventricular dysfunction [44]. As shown in our results, the plasma levels of cTnI, NT-proBNP, and CRP were lower in patients after restricting volumes of resuscitation fluid strategy with intravenous infusion of UTI than in those after restricting volumes of resuscitation fluid strategy alone.

The concentration of blood LA has been considered as an indicator of tissue perfusion changes in critically ill patients [45]. Some research studies indicated that the blood LA concentrations in the nonsurvivor group were higher than those in the survivor group [46–48]. Abnormal coagulation is one of the manifestations in sepsis [49], and several studies have indirectly demonstrated that coagulation function was impaired in patients with sepsis [50, 51]. This study indicated that the concentration of blood LA was lower in the UTI group, and the PT and PATT were superior to those in restrictive fluid resuscitation without UTI. Acute renal failure commonly occurs with severe sepsis and is associated with high mortality [52]. An early marker of acute renal failure could impact on the management of such patients. Renal dysfunction is assessed by increases in levels of BUN, Cr, and UA. In our study, reduced levels of BUN, Cr, and UA were determined in patients after restricting volumes of resuscitation fluid strategy with intravenous infusion of UTI compared with those after restricting volumes of resuscitation fluid strategy alone.

Taken together, the findings obtained from our results support the notion that UTI as an adjuvant therapy for restricting volumes of resuscitation fluid strategy in treating septic shock may decrease the LA level, attenuate inflammatory edema, reduce vascular permeability, prevent pulmonary edema, and restore cardiac and renal functions. The outcomes in our study might change a little bit due to the small number of included patients and the shorter observation time. Therefore, further investigations with a large cohort of patients with septic shock are required.

## Figures and Tables

**Figure 1:** The plasma levels of cTnI, NT-proBNP, and CRP in patients with septic shock before and after restricting volumes of resuscitation fluid strategy with or without intravenous infusion of UTI. The letter a indicates *P* < 0.05 compared to pretreatment, and b indicates *P* < 0.05 compared to the fluid restriction group.

**Figure 2:** The volume of 24 h urine and the levels of BUN, Cr, and UA in patients with septic shock before and after restricting volumes of resuscitation fluid strategy with or without intravenous infusion of UTI. The letter a indicates *P* < 0.05 compared to pretreatment, and b indicates *P* < 0.05 compared to the fluid restriction group.

**Table 1:** Comparison of baseline variables by group.

Variable	Fluid restriction + UTI (*n* = 89)	Fluid restriction (*n* = 93)	*P*
Sex, male no. (%)	61 (68.54%)	65 (69.90%)	0.843
Age, year	62.24 ± 14.83	60.52 ± 11.71	0.385

Source of sepsis, no. (%)			0.995
Lung	27 (30.34%)	29 (31.18%)	
Chest	26 (29.21%)	27 (29.03%)	
Abdomen	22 (24.47%)	23 (24.73%)	
Soft tissue	10 (11.24%)	11 (11.83%)	
Others	4 (4.49%)	3 (3.23%)	

**Table 2:** The changes of SVRI, PVPI, and EVLWI in patients with septic shock before and after restricting volumes of resuscitation fluid strategy with or without intravenous infusion of UTI.

Group	Case	SVRI (dyn·s·cm^−5^·m^2^)		PVPI (dyn·s·cm^−5^·m^2^)		EVLWI (ml/kg)	
		Before treatment	After treatment	Before treatment	After treatment	Before treatment	After treatment
Fluid restriction + UTI	89	981 ± 154	1465 ± 359^a^	5.08 ± 1.36	2.51 ± 0.65^a^	9.22 ± 2.87	5.63 ± 1.59^a^
Fluid restriction	93	995 ± 168	1253 ± 317^a^	4.93 ± 1.42	3.90 ± 0.72^a^	9.17 ± 2.80	7.75 ± 2.01^a^
*t*	—	0.585	4.199	0.727	13.650	0.119	7.869
*P*	—	0.559	<0.001	0.468	<0.001	0.905	<0.001

The letter a indicates *P* < 0.05 compared to pretreatment. SVRI: systemic vascular resistance index; EVLWI: extravascular lung water index; PVPI: pulmonary vascular permeability index.

**Table 3:** The cardiac function of patients with septic shock before and after restricting volumes of resuscitation fluid strategy with or without intravenous infusion of UTI.

Index	Fluid restriction + UTI (*n* = 89)	Fluid restriction (*n* = 93)	*t*	*P*
MAP (mmHg)				
Before treatment	50.21 ± 5.22	51.07 ± 4.95	1.141	0.256
After treatment	82.84 ± 3.93^a^	74.44 ± 5.16^a^	12.31	<0.001

CO (L/min)				
Before treatment	4.32 ± 1.41	4.27 ± 1.35	0.244	0.807
After treatment	5.40 ± 1.52^a^	4.91 ± 1.44^a^	2.233	0.027

LVEF (%)				
Before treatment	37.83 ± 9.48	38.42 ± 10.75	0.392	0.695
After treatment	47.34 ± 8.92^a^	42.59 ± 9.07^a^	3.56	<0.001

SV (ml)				
Before treatment	64.58 ± 11.47	64.62 ± 10.91	0.024	0.981
After treatment	76.93 ± 12.65^a^	71.62 ± 12.04^a^	2.901	0.004

HR (time/min)				
Before treatment	122.80 ± 10.14	124.14 ± 13.09	0.770	0.443
After treatment	81.25 ± 8.14^a^	88.46 ± 6.92^a^	6.448	<0.001

The letter a indicates *P* < 0.05 compared to pretreatment; MAP: mean artery pressure; CO: cardiac output; LVEF: left ventricular ejection fraction; SV: stroke volume; HR: heart rate.

**Table 4:** The LA and coagulation function of patients with septic shock before and after restricting volumes of resuscitation fluid strategy with or without intravenous infusion of UTI.

Group	Case	LA level (mmol/L)		PT (s)		PATT (s)	
		Before treatment	After treatment	Before treatment	After treatment	Before treatment	After treatment
Fluid restriction ± UTI	89	15.12 ± 3.05	3.97 ± 0.63^a^	9.82 ± 1.20	11.24 ± 1.38^a^	28.43 ± 4.47	32.73 ± 4.29^a^
Fluid restriction	93	15.23 ± 2.74	6.25 ± 0.94^a^	9.64 ± 1.32	15.49 ± 1.29^a^	28.35 ± 4.50	39.28 ± 3.52^a^
*t*	—	0.069	19.140	0.961	21.470	0.120	11.140
*P*	—	0.945	<0.001	0.338	<0.001	0.904	<0.001

The letter a indicates *P* < 0.05 compared to pretreatment; PT: prothrombin time; PATT: partially activated thrombin time.

**Table 5:** The APACHE II and SOFA scores of patients with septic shock before and after restricting volumes of resuscitation fluid strategy with or without intravenous infusion of UTI.

Group	Case	APACHE II scores		SOFA scores	
		Before treatment	After treatment	Before treatment	After treatment
Fluid restriction + UTI	89	29.57 ± 4.23	11.42 ± 2.38^a^	13.78 ± 2.73	4.67 ± 1.51^a^
Fluid restriction	93	28.66 ± 4.11	15.46 ± 3.08^a^	13.44 ± 3.52	6.79 ± 2.08^a^
*t*	—	1.472	2.438	0.726	7.839
*P*	—	0.143	0.016	0.469	<0.001

The letter a indicates *P* < 0.05 compared to pretreatment; APACHE II: Acute Physiology and Chronic Health Evaluation; SOFA: sequential organ failure assessment.

**Table 6:** The mortality of patients with septic shock after restricting volumes of resuscitation fluid strategy with or without intravenous infusion of UTI.

Group	Case	Mortality (%)
Fluid restriction + UTI	89	25 (28.09)
Fluid restriction	93	28 (30.11)
*Z*	—	0.299
*P*	—	0.765

## Data Availability

The data used to support the findings of this study are included within the article.
